This article has been retracted.

# Clinical Efficacy of Retroauricular Injection of Methylprednisolone Sodium Succinate in the Treatment of Sudden Deafness with Type 2 Diabetes

**DOI:** 10.1155/2022/3097436

**Published:** 2022-07-22

**Authors:** Zhenbo Zhong, Xiaofei Wang, Kairui Xu, Jing Tao

**Affiliations:** Department of Otolaryngology, Lishui People's Hospital, Lishui, 323000 Zhejiang Province, China

## Abstract

**Background:**

The etiology of sudden deafness is still unclear. In recent years, people's life rhythm is getting faster and faster. Fatigue, environment, diet, psychology, and other factors have increased the morbidity rate of sudden deafness and improved the quality of life of patients. And work efficiency is greatly affected.

**Aims:**

A study to investigate the clinical efficacy of postauricular injection of methylprednisolone sodium succinate in the treatment of sudden deafness with type 2 diabetes.

**Materials and Methods:**

Sixty patients with sudden deafness who were treated in our hospital from January 2018 to October 2020 were selected as the subjects of this prospective study and divided into 30 cases each in the comparison group and the observation group according to the random number remainder grouping method. The comparison group was treated conventionally, and the observation group was treated with postauricular injection of methylprednisolone sodium succinate on the basis of the comparison group. Patients in the two groups were observed and compared on the 3rd, 6th, and 9th days after treatment with pure-tone hearing threshold checks and regular monitoring of blood glucose, blood rheology, and other indexes.

**Results:**

On the 7th, 14th, and 30th days after treatment, the pure-tone audiometric thresholds of the two groups were gradually decreased, and the changes in the pure-tone audiometric thresholds in the observation group were greater than those in the control group. After lunch on the 6th day and after lunch on the 9th day, it was lower than that in the control group, and the difference was statistically significant (*P* < 0.05). 30 days after treatment, the blood viscosity, fibrin, and platelet aggregation rate of the observation group were significantly lower than those of the control group. After treatment, the clinical efficacy rate of the observation group was 96%, which was significantly higher than that of the control group, 80%, and the above differences were statistically significant (*P* < 0.05).

**Conclusion:**

Treatment with postauricular injection of methylprednisolone sodium succinate has shown better therapeutic recovery in patients with sudden deafness, improved pure-tone hearing threshold, reduced risk of blood glucose elevation, and improved clinical outcomes for patients with sudden deafness, providing some reference for the treatment of patients with sudden deafness.

## 1. Introduction

Sudden deafness is a sudden onset of unexplained sensorineural hearing loss within 72 hours, with hearing loss in at least two adjacent frequencies [1]. Type 2 diabetes patients are more likely to develop sudden deafness due to their own disease characteristics. Currently, it is believed that diabetes causes sudden deafness, and statistics show that the proportion of sudden deafness with type 2 diabetes is 15% [2]. Because of the side effects of systemic application of hormones, hormone therapy was abandoned in the past for such patients, resulting in a greatly reduced efficacy [2]. Methylprednisolone sodium succinate is a synthetic glucocorticoid with strong anti-inflammatory, immunosuppressive, and antiallergic activities. Glucocorticoids diffuse across cell membranes and bind to specific receptors in the cytoplasm.

The etiology of sudden deafness is still unclear. In recent years, people's lives have become increasingly fast-paced, and fatigue and environmental, dietary, and psychological factors have increased the incidence of sudden deafness, causing a greater impact on patients' quality of life and work efficiency [3]. Despite prompt treatment, some patients still suffer from permanent hearing loss and tinnitus, which is a serious otologic disease that endangers human health [4]. It is therefore the responsibility of medical professionals to find effective treatments for sudden deafness with few safe side effects [5]. In particular, for patients with sudden deafness whose diabetes is aggravated by the application of hormones, it is particularly important to choose an appropriate treatment plan, considering the effectiveness of hormones in the treatment of sudden deafness and the intolerance of type 2 diabetic patients to the systemic use of glucocorticoids [6]. The use of retroauricular injection of methylprednisolone sodium succinate as a treatment option for patients with sudden deafness with type 2 diabetes can solve a practical problem in current clinical work.

## 2. Material and Methods

### 2.1. Research Object

All records of the identity of the patients included in our study who underwent treatment in our hospital from January 2018 to October 2020 will be kept in the hospital as required, and all records regarding the identity of the patients will not be disclosed in the public report of the study results. Patients will give informed consent prior to enrollment; communicate fully with patients before the experiment; introduce the content and process of the experiment, the associated risks, and possible adverse effects; sign the informed consent form after obtaining patients' consent, and inform patients of the test results in strict accordance with the standard operation of the experimental procedure. The sample size was calculated based on the cross-sectional survey sample size formula: *n* = *t*_*a*_^2^*PQ*/*d*^2^, where *n* is the sample size, *P* is the prevalence of sudden onset deafness, *Q* = 1 − *P*, *d* is the permissible error, *a* = 0.05, and *t*_*a*_ = 1.96. The minimum sample size was 57 cases, and the actual sample size of our study was 60 cases. The cases were divided into a comparison group and an observation group of 30 cases each according to the random number residual grouping method. Diagnostic criteria [7]: sudden sensorineural hearing loss occurring within three days, with hearing loss ≥ 20 dB at least at two adjacent frequencies, mostly in one ear, but in a few cases it may occur bilaterally or sequentially; no clear causative factor was found; it may be accompanied by ear symptoms such as tinnitus and a sense of ear stuffiness; it may be accompanied by systemic manifestations such as vertigo, nausea, and vomiting.

### 2.2. Inclusion and Exclusion Criteria

Case selection criteria: (i) age between 18 and 70 years, regardless of gender; (ii) patients were enrolled with unilateral deafness, routine otologic examination to exclude external ear, middle ear disease and deafness caused by the central nervous system, and the onset of deafness was between 1 day and 2 weeks; (iii) diagnosis of type 2 diabetes mellitus was confirmed; (iv) routine otologic examination and related tests excluded deafness due to external ear, middle ear, central nervous system, and trauma, and all enrolled patients met the diagnostic criteria for sudden deafness established by the Chinese Medical Association, Otolaryngology Branch. Patients did not receive any related treatment before admission. The possible adverse effects of topical application of hormones and the reasons for using them as the preferred treatment were clearly communicated, and all patients were asked to sign an informed consent form. Exclusion criteria: (i) more than 1 week from onset to consultation, cranial nao lesions other than the V VIII pair of cerebral nerves, organic lesions in the external, middle, and inner ear found on admission examination; (ii) patients with primary diseases such as digestive and hematological system other than hypertension and diabetes, pregnant and lactating women, and patients diagnosed with psychiatric disorders; (iii) patients who do not cooperate with the treatment affecting the progress of the experiment and the observation of the efficacy.

## 3. Methods

Both groups of patients underwent pure-tone hearing threshold examination and liver and kidney function and routine blood and urine examinations before and after treatment. The control group was given conventional treatments such as reducing fibrinogen, improving inner ear microcirculation, and nourishing nerves and microwaves, including nails. Cobalamin (manufactured by Harbin Sanlian Pharmaceutical Co., Ltd., approved by Chinese medicine H20044627, specification: 1 ml/0.5 mg) 0.5 mg times + vitamin B1 injection (produced by Sinopharm Rongsheng Pharmaceutical Co., Ltd., approved by Chinese medicine H41020100, specification: 2 ml/100 mg) 100 mg, followed by intramuscular injection, 1 time/d. Add 25 ml of ginkgo biloba extract injection into 500 ml of 0.9% sodium chloride solution for intravenous drip, once a day. Observation group: mix 40 mg of methylprednisolone sodium succinate (national medicine approved word: H20080284, Tianjin Tianan Pharmaceutical Co., Ltd., specification: 40 mg/ml) with 1 ml of 0.9% sodium chloride solution, and then, prepare 2 ml of mixed solution. At the level of the upper border of the external auditory canal, the subperiosteal area of the mastoid and the 8-10 mm postauricular hook are injected for treatment, once every other day, for a total of 3 to 5 times, of which the subperiosteal area is the acupuncture site, and continuous compression is performed for 6 minutes after the injection.

### 3.1. Observation Index

The level of air conduction hearing threshold was obtained by pure-tone audiometry, the test must be conducted in a standard soundproof room with bottom noise < 25 dB(A), the equipment must be calibrated by the relevant professional structure before use, and the pure-tone hearing threshold test was conducted in accordance with the national GB/T16403-1996 standard; the air conduction threshold is the degree of hearing impairment; the higher it is, the more hearing impairment. The Simple Coping Scale (SCSQ) was used to assess 20 items, including two dimensions of positive coping (12 items) and negative coping (8 items), and the options were divided into four levels of “no, occasionally, sometimes, and often,” with scores of 0~3. The higher the score, the more frequently it was used. The efficacy criteria: healed: the damaged frequency hearing returned to normal, or up to the level of the healthy ear, or up to the level before the disease; effective: the damaged frequency average hearing improved by more than 30 dB; effective: the damaged frequency average hearing improved by 15-30 dB; ineffective: the damaged frequency average hearing improved by less than 15 dB. The scale was independent of age, gender, and economic status, and Cronbach's *α* value was greater than 0.914 before use. Before treatment and after lunch on the 3rd day, after lunch on the 6th day, and after lunch on the 9th day, blood was drawn to detect blood sugar.

### 3.2. Statistical Analysis

All statistical data in this study were entered into Excel software by the first author and the corresponding author, respectively, and the statistical processing software was SPSS 25.0 for calculation. Repeated measures analysis of variance between groups was used to measure the measurement expressed as mean ± standard deviation (*X* ± *S*). Count data expressed as a percentage (%) were tested by *χ*^2^. Univariate and logistic multivariate regression analysis was used to compare the influencing factors, and the risk factors with significant differences were screened. Correlation test used logistic regression linear correlation analysis. Included data that did not conform to a normal distribution were described by *M*(*QR*), using the Mann–Whitney test.

## 4. Results

### 4.1. Comparison of Baseline Data

There was no statistically significant difference in mean age, gender, mean disease duration, body mass index, and side between the two groups (*P* > 0.05). See Table 1.

### 4.2. Pure-Tone Hearing Threshold Examination Comparison

Before treatment, there was no statistically significant difference between the two groups in the pure-tone hearing threshold examination (*P* > 0.05). After treatment, the pure-tone hearing threshold examination was gradually reduced in both groups on days 7, 14, and 30, and the degree of change in the pure-tone hearing threshold index was greater in the observation group than in the comparison group, and the differences were statistically significant (*P* < 0.05). See Figure 1.

### 4.3. Comparison of Blood Glucose

Before treatment, there was no statistically significant difference in the comparison of blood glucose between the two groups (*P* > 0.05). After treatment, patients in the observation group showed an increase in blood glucose after lunch on days 3, 6, and 9 compared to the control group, but the difference was not statistically significant (*P* > 0.05). See Figure 2.

### 4.4. Comparison of Rheological Parameters

Before treatment, there was no significant difference in the hemorheological indexes between the two groups (*P* > 0.05). Thirty days after treatment, the blood viscosity, fibrin, and platelet aggregation rate of the observation group were significantly lower than those of the control group, with statistical significance (*P* < 0.05). See Figure 3.

### 4.5. Comparison of Clinical Efficacy

After treatment, the clinical efficacy rate of the observation group was 96%, which was significantly higher than that of the control group, 80%, and the difference was statistically significant (*P* < 0.05). See Figure 4.

## 5. Discussion

It is clinically believed that the occurrence of sudden deafness is triggered by impaired blood supply to the inner ear, high blood viscosity, and vascular endothelial dysfunction, in addition to the inflammatory state of the cochlea [8]. According to the anatomy of the ear, the internal auditory artery and the vagus artery are the main arteries supplying the inner ear, which are supplied by the anterior or posterior inferior cerebellar artery and the vertebrobasilar artery, respectively, while the middle and outer ear is supplied by the carotid artery system [9]. When the arteries supplying the inner ear suffer from vascular occlusion vascular stenosis or vascular sclerosis, it is easy to cause impairment of inner ear blood supply. If the collateral circulation is not established in time, it will lead to severe hypoxia and ischemia in the inner ear [10]. Clinical studies have found that patients with sudden deafness also have varying degrees of abnormal blood rheology indicators, suggesting that the erythrocyte deformation index in the blood shows increased characteristics [11]. The increased viscosity of the blood allows a large number of platelets to coagulate, which leads to a constant state of hypercoagulation [12]. In a hypercoagulable state, ischemia and hypoxia in the inner ear become more and more severe, and the oxygen demand of cochlear cells gradually increases, which can easily lead to vascular embolism, spasm, and sclerosis and also cause metabolic disorders, which then damage the sensory nerve endings and cause dizziness and tinnitus and hearing loss [13]. Therefore, the treatment of sudden deafness should be integrated with the characteristics of its pathogenesis to take targeted therapeutic measures.

We study that postauricular injection is a new and more direct and effective drug delivery method carried out in recent years [14], which can avoid the blood-vagus barrier and enter the inner ear directly so that the internal and external lymphatic fluid can obtain higher drug concentrations, while avoiding the disadvantages of the drum chamber administration of drug concentration is not easy to control and the efficacy is unstable [15]. From the anatomical point of view, blood in the retroauricular region first returns to the retroauricular vein, and then, part of it converges via the mastoid conduit vein into the sigmoid sinus, which is adjacent to the distal endolymphatic sac, and the connective tissue between them is tightly bound [16]. The drug injected behind the ear can quickly reach the sigmoid sinus through the retroauricular vein and the mastoid vein and then diffuse to the endolymphatic sac, maintain a high concentration, and then reflux to the inner ear through the microvenules around the endolymphatic sac to achieve an effective therapeutic concentration to exert pharmacological effects [17]. Currently, all relevant studies in China have confirmed the effectiveness of postauricular injection of glucocorticoids in the treatment of all types of sudden deafness [18], and this new mode of drug delivery will be the future trend in the standardized treatment of sudden deafness.

We studied patients treated with postauricular injection of sodium methylprednisolone succinate and analyzed its specific mechanism of action as follows: an appropriate amount of the drug was given to be injected into the subpapillary area of the patient's mastoid bone, in which the drug was absorbed by the body through local infiltration and the mastoid bone could be in close contact with the mastoid periosteum. The absorption rate after local administration is reduced to prevent the drug from spreading to the whole body and to reduce the adverse effects caused by systemic administration [19]. The osmolarity gradient can be based on the blood-vagus barrier and the blood-exolymphatic barrier into the human exolymphatic fluid, helping patients to establish an osmotic gradient of internal and external lymphatic fluid, facilitating the effective improvement of endolymphatic dehydration symptoms and achieving good immunosuppressive and antivertigo efficacy, making the patients' inner ear microcirculation and inner ear hair cell status to be effectively improved [20].

In our study, 30 days after treatment, the blood viscosity, fibrin, and platelet coagulation rates of patients in the observation group were significantly lower than those in the comparison group, indicating that the treatment with injectable methylprednisolone sodium succinate combined with ginkgo biloba could effectively regulate the rheological indexes and promote the improvement of their inner ear blood circulation. Methylprednisolone sodium succinate is an injectable glucocorticoid drug that can bind to specific receptors in the cytoplasm through the cell membrane and subsequently enter the nucleus to bind to DNA and initiate transcription of mRNA, which in turn synthesizes various proteases [21]. The drug has a strong anti-inflammatory effect, inhibits the proliferation of bacteria or viruses in the cochlea, and effectively reduces the inflammatory response of the cochlea. It also has certain neuroprotective functions, which can relieve the symptoms of neuroedema, promote the improvement of microcirculation in the ear, and keep the lymphatic fluid in the ear in a balanced state thus further relieving the symptoms of sudden deafness, tinnitus, and vertigo and making their hearing improve [22]. Although injectable methylprednisolone sodium succinate has a good effect in reducing the inflammatory response of the cochlea, it does not improve the impaired blood supply to the inner ear or reduce the blood viscosity [23]. Ginkgo biloba extract, the main component of ginkgo biloba tablets, contains flavonol glycosides, endolipids, and amino acids, which also have the same effect as injectable methylprednisolone sodium succinate in eliminating the persistent inflammatory state of the cochlea and improving the cochlear nerve nutrient supply, thus reducing the degree of hearing impairment in sudden deafness [24]. The addition of ginkgo biloba to the anti-inflammatory treatment with the glucocorticoid drug methylprednisolone sodium succinate can eliminate the cochlear inflammatory response as much as possible and maximize the improvement of cochlear blood circulation, thus reducing the degree of hearing impairment and promoting rapid recovery of their hearing [25].

In our study, for patients with sudden deafness accompanied by type 2 diabetes, this mode of administration may lead to aggravation of diabetes, and some patients may even develop serious complications such as diabetic ketoacidosis, making diabetes a relative contraindication to glucocorticoid use. To address this problem, local injection of hormones has become a possible option, which can increase the drug concentration in the inner ear, reduce the amount of hormones, and decrease the effect on systemic blood glucose concentrations compared with systemic administration, thus providing higher efficacy and safety [26]. Some studies have demonstrated that methylprednisolone sodium succinate has the highest local concentration and neuroprotective effects compared to other commonly used glucocorticoids [27]. Methylprednisolone is an intermediate-acting glucocorticoid with a high rate of intraplasma metabolism and intracellular activity, which persists intracellularly even when undetectable in the plasma [28]. Therefore, it is used in the treatment of sudden deafness by local injection. Subperiosteal injection administration behind the ear and tympanic ventricular injection administration are both localized [29]. Transvocal drug delivery is characterized by drug absorption through the tympanic chamber via the round window, and this mode of drug delivery bypasses the blood-vagus barrier, allowing the drug to bind directly to the inner ear hormone receptors and act [30]. This results in higher local drug concentrations in the inner ear and lower drug concentrations in the systemic circulation, thus reducing the effect of hormones on fluctuations in blood glucose concentrations.

Our study is a small sample trial, and in the future, conditions allow for a large sample, multicenter clinical study to make the clinical efficacy observation results more convincing and provide a safe and effective method for the treatment of patients with sudden deafness combined with diabetes mellitus, which can be used to guide clinical treatment. The etiology and pathogenesis of sudden deafness are complex and unclear. The clinical efficacy of postauricular steroid hormone injections in patients with sudden deafness who have contraindications to hormones is better than other hormone applications, and the side effects are less, so it can be used as the preferred treatment for patients with sudden deafness who have contraindications to glucocorticoids in the future. It may be the first choice of treatment for patients with sudden deafness who have contraindications to glucocorticoids in the future and may bring benefits to patients with sudden deafness in combination with diabetes.

In conclusion, postauricular injection of methylprednisolone sodium succinate has a low glycemic impact and no systemic adverse effects were observed. The postauricular injection of methylprednisolone sodium succinate is clinically effective, simple, safe, and reliable, without toxic side effects, easily accepted by patients and their families, with good patient compliance and few side effects, and provides a reference for the treatment of patients with sudden deafness.

## Figures and Tables

**Figure 1:** Comparison of pure-tone audiometry between two groups of patients. In this study, the pure-tone hearing threshold statistics of the two groups of patients were input into Excel software by the first author and the corresponding author, respectively, and the Shapiro-Wilk method of mean ± standard deviation was used for inclusion test. ANOVA was performed between groups to find out. On the 3rd, 6th, and 9th days after treatment, the pure-tone hearing thresholds of the two groups were gradually decreased, and the changes of the pure-tone hearing thresholds in the observation group were greater than those in the control group. The difference is not statistically significant (*P* > 0.05).

**Figure 2:** Blood sugar comparison. Statistics for blood glucose comparisons in this study were entered into Excel software by the first and corresponding authors, respectively, and indicators were included in the test using the Shapiro-Wilk method of mean ± standard deviation. And independent sample or paired sample *t*-test was implemented between groups found. Patients in the observation group showed an increase in blood glucose after lunch on days 3, 6, and 9 compared to the control group, but the difference was not statistically significant (*P* > 0.05).

**Figure 3:** Comparison of rheological parameters. In this study, the statistics of the rheological indexes of the two groups of patients were input into Excel software by the first author and the corresponding author, respectively, and the indexes such as blood viscosity, fibrin, and platelet aggregation rate were included in the test using the Shapiro-Wilk method of mean ± standard deviation. Independent samples or paired samples *t*-tests were performed between groups or within groups to find out. Before treatment, there was no significant difference in the hemorheological indexes between the two groups (*P* > 0.05). 30 days after treatment, the (a) blood viscosity, (b) fibrin, and (c) platelet aggregation rate in the observation group were significantly lower than those in the control group, with statistical significance (*P* < 0.05).

**Figure 4:** Comparison of clinical efficacy. In this study, the statistics of the clinical efficacy of the two groups of patients were input into Excel software by the first author and the corresponding author, respectively, and the data were expressed as integers and found by the chi-square test. After treatment, the clinical efficacy rate of patients in the observation group was 96%, which was significantly higher than that in the control group, 80%, with statistical significance (*P* < 0.05).

**Table 1:** Comparison of baseline information of patients in the two groups.

Group	Average age (years)	Gender (male/female)	Average duration of illness (day)	Body mass index (kg/m^2^)	Side (*N*)	
					Left	Right
Comparison group (30)	59.83 ± 2.13	13/17	8.12 ± 1.16	29.32 ± 2.16	12	18
Observation group (30)	58.72 ± 3.16	16/14	7.91 ± 1.10	29.11 ± 1.10	17	13
*t*/*x*^2^	1.595	0.601	0.720	0.203	1.669	
*P*	0.116	0.438	0.475	0.840	0.196	

## Data Availability

The simulation experiment data used to support the findings of this study are available from the corresponding author upon request.

## References

[1] Shao M., Xiong G., Xiang G., Xu S., Zheng Y., Zhang L. (2021). Sudden deafness as an initial presentation of varicella: case report and literature review. *Annals of Palliative Medicine*.

[2] Herrera M., García Berrocal J. R., García Arumí A., Lavilla M. J., Plaza G. (2019). Grupo de Trabajo de la Comisión de Audiología de la SEORL. Update on consensus on diagnosis and treatment of idiopathic sudden sensorineural hearing loss. *Acta Otorrinolaringológica Española*.

[3] Si J. P., Jiang H., Li Y. Y. (2020). Correlation between effectual time and the curative effect in patients with all frequency descending sudden deafness after treatment. *American Journal of Otolaryngology*.

[4] Peng C., Lei J. X. (2020). Compatible stability of methylprednisolone sodium succinate and tropisetron in 0.9% sodium chloride injection. *European Journal of Hospital Pharmacy*.

[5] Lu H. Y., Wang R. Q., Li X., Li X. (2020). Pharmacokinetics after periocular methylprednisolone sodium succinate injection in rabbit eyes. *Evidence-Based Complementary and Alternative Medicine*.

[6] Kuhn M., Heman-Ackah S. E., Shaikh J. A., Roehm P. C. (2011). Sudden sensorineural hearing loss: a review of diagnosis, treatment, and prognosis. *Trends in Amplification*.

[7] Cottrell J., Zahr S. K., Yip J. (2021). Quality indicators for the diagnosis and management of sudden sensorineural hearing loss. *Otology & Neurotology*.

[8] Lee H., Baloh R. W. (2005). Sudden deafness in vertebrobasilar ischemia: clinical features, vascular topographical patterns and long-term outcome. *Journal of the Neurological Sciences*.

[9] Blasco M. A., Redleaf M. I. (2014). Cochlear implantation in unilateral sudden deafness improves tinnitus and speech comprehension: meta-analysis and systematic review. *Otology & Neurotology*.

[10] Chen Y. C., Tsai S. J., Chen J. C., Hwang J. H. (2019). Risks of tinnitus, sensorineural hearing impairment, and sudden deafness in patients with non-migraine headache. *PLoS One*.

[11] Qiao S., Duan L., Luo S., Fan G. J. (2019). Intractable sudden deafness treated with acupuncture on the base of “heart housing the mind”. *Zhongguo Zhen jiu= Chinese Acupuncture & Moxibustion*.

[12] Young Y. H. (2020). Contemporary review of the causes and differential diagnosis of sudden sensorineural hearing loss. *International Journal of Audiology*.

[13] Herrera M., García Berrocal J. R., García Arumí A., Lavilla M. J., Plaza G., Grupo de Trabajo de la Comisión de Audiología de la SEORL (2019). Update on consensus on diagnosis and treatment of idiopathic sudden sensorineural hearing loss. *Acta Otorrinolaringologica (English Edition)*.

[14] Yang X., Yu L., Ma X. (2007). Postauricular injection of compound betamethasone in the treatment of intractable low-frequency sensorineural hearing loss. *Chinese Journal of Otolaryngology Head and Neck Surgery*.

[15] Li K., Yu L., Xia R. (2012). 7.0T magnetic resonance imaging to observe the feasibility of post-auricular administration to promote drug entry into the inner ear. *Chinese Journal of Otology*.

[16] Wang F., Xuemei L., Zhu Y. (2015). Efficacy analysis of post-auricular medication in the treatment of mid-high frequency descending sudden hearing loss. *Journal of Clinical Otolaryngology Head and Neck Surgery*.

[17] Li X., Zhang X. Y., Wang Q. J., Wang D. Y. (2015). Efficacy of methylprednisolone sodium succinate for injection (postotic injection) on the auditory threshold and speech recognition rate of sudden deafness patients. *International Journal of Clinical and Experimental Medicine*.

[18] Amano H., Kitagawa Y., Hayakawa T., Muto T., Okumura A., Iwayama H. (2021). Methylprednisolone-induced anaphylaxis diagnosed by intradermal skin test: a case report. *Allergy, Asthma & Clinical Immunology*.

[19] Caruso M. C., Daugherty M. C., Moody S. M., Falcone R. A., Bierbrauer K. S., Geis G. L. (2017). Lessons learned from administration of high-dose methylprednisolone sodium succinate for acute pediatric spinal cord injuries. *Journal of Neurosurgery. Pediatrics*.

[20] Karabey-Akyurek Y., Gurcay A. G., Gurcan O. (2017). Localized delivery of methylprednisolone sodium succinate with polymeric nanoparticles in experimental injured spinal cord model. *Pharmaceutical Development and Technology*.

[21] Levy Y., Segal N., Nahum A., Marcus N., Garty B. Z. (2014). Hypersensitivity to methylprednisolone sodium succinate in children with milk allergy. *The Journal of Allergy and Clinical Immunology. In Practice*.

[22] Xu F., Feng E., Su L., Xu G. (2013). Doxofylline and methylprednisolone sodium succinate are stable and compatible under normal injection conditions. *Pakistan Journal of Pharmaceutical Sciences*.

[23] Igneri L. A., Czosnowski Q. A., Whitman C. B. (2013). Methylprednisolone sodium succinate-associated macroglossia in a critically ill patient. *Pharmacotherapy*.

[24] D’Hondt M., Vangheluwe E., Van Dorpe S. (2012). Stability of extemporaneously prepared cytarabine, methotrexate sodium, and methylprednisolone sodium succinate. *American Journal of Health-System Pharmacy*.

[25] Nishida H., Tanaka H., Kitamura M., Inaba T., Nakayama M. (2016). Methylprednisolone sodium succinate reduces spinal cord swelling but does not affect recovery of dogs with surgically treated thoracolumbar intervertebral disk herniation. *The Japanese Journal of Veterinary Research*.

[26] Cheng S., Gao W., Xu X. (2016). Methylprednisolone sodium succinate reduces BBB disruption and inflammation in a model mouse of intracranial haemorrhage. *Brain Research Bulletin*.

[27] Wang W., Zuo B., Liu H., Cui L. (2019). Intermittent injection of methylprednisolone sodium succinate in the treatment of cervical spinal cord injury complicated with incomplete paraplegia. *Pakistan Journal of Medical Sciences*.

[28] Jie C., Li-Po H., Yu Z., Yuan-da Z. (2020). Effectiveness of gamma globulin combined with methylprednisolone sodium succinate in severe hand foot mouth disease - Baoding Children’s Hospital, China. *JPMA. The Journal of the Pakistan Medical Association*.

[29] Ren G., Xu J., Lan L., Ma B., Zhang Q. (2021). Postauricular injection of methylprednisolone sodium succinate as a salvage treatment for refractory sudden sensorineural hearing loss. *Irish Journal of Medical Science*.

[30] Wang D. L., Song H. D., Hao Q. P. (2021). Application of methylprednisolone sodium succinate combined with tropisetron in prevention of nausea and vomiting under microvascular decompression of hemifacial spasm. *Zhongguo yi xue ke xue Yuan xue bao. Acta Academiae Medicinae Sinicae*.

